# Performance Optimization of Surface Plasmon Resonance Imaging Sensor Network Based on the Multi-Objective Optimization Algorithm

**DOI:** 10.1155/2022/3692984

**Published:** 2022-07-31

**Authors:** Zhiyou Wang, Maojin Wang, Ying Chen, Fangrong Hu

**Affiliations:** ^1^School of Electronic Communication and Electrical Engineering, Changsha University, Kaifu District, Changsha, China; ^2^Hunan Engineering Technology Research Center of Optoelectronic Health Detection, Changsha, China; ^3^Guangxi Key Laboratory of Automatic Detecting Technology and Instrument, Guilin University of Electronic Technology, Guilin 541004, China

## Abstract

In this work, we report performance optimization of a wireless sensor network (WSN) based on the plain silver surface plasmon resonance imaging (SPRi) sensor. At the sensor node level, we established the refractive index-thickness models for both gold and silver in the sensor and calculated the depth-width ratio (DWR) and penetration depth (PD) values of the sensor of different gold and silver thicknesses by the Jones transfer matrix and Kriging interpolation. We optimized the DWR and PD simultaneously by using the multi-objective optimization genetic algorithm (MOGA). In the following performance optimization of WSN, we simultaneously optimized the transmission success rate and information dimension with the number of nodes and transmission failure rate of the sensor node as variables by the same algorithm. By calculating the information dimension and the transmission success rate of each Pareto optimal solution, we obtained the number of nodes and transmission failure probability of the node available for practical deployment of WSN. The above results indicate that the Pareto optimal solution set obtained from MOGA can help to provide the best solution for the optimization of some certain performance parameters and also assist us in making the trade-off decision in the structure design and network deployment if optimal values of all the performance parameters can be obtained simultaneously.

## 1. Introduction

Surface plasmon resonance imaging (SPRi) detection is one type of label-free and contact-free assays which do not alter or impair the function of biomolecules. Because of its ability to acquire the endpoint signal and binding intensity information simultaneously during drug screening and protein sequencing, the SPRi technique has been widely applied in cancer immunotherapy, drug development, food safety, and other important fields [1–4]. To achieve further applications in early diagnosis and point of care testing (POCT) cases, the performances of the SPRi sensors need to be promoted in the following ways. First, the sensors should be configured as miniaturized devices of high detection sensitivity in mobile and noisy scenes. Among varieties of metals in the SPRi configuration, gold and silver have been the main choices in the reported works [5–7]. Compared with gold film-based SPRi sensors, silver film-based sensors demonstrated around 1-time sensitivity enhancement. Although the chemical properties of silver are more active than gold, the reported plain silver SPRi sensors prepared by using a gold island film as the adhesion enhancing layer between the silver film and the chromium adhesion layer show the same level of stability as the gold thin film-based sensors. The working life of plain silver SPRi sensors can reach more than 8 hours in chemical reagents such as strong acids, strong bases, and highly permeable salt solutions [8, 9]. To further improve the sensitivity performance of the plain silver SPRi sensor, two factors need to be considered comprehensively. The first is the depth-width ratio (DWR), which is defined as the ratio between the depth and full width at half maximum (FWHM) of the SPR curve. According to Homola et al. work, the SPRi sensors with higher DWR values feature higher sensitivity and lower resolution in detection [10]. The second is evanescent wave penetration depth (PD) into the measured biomolecules, which is defined as the distance from the silver surface where the electromagnetic field intensity drops to 1/*e*^2^ of the value at the surface. In our previous work, a larger PD value was reported to be helpful for the detection of weak binding signals between biomolecules at the immobilized cell surface [8]. Second, the SPRi sensors should be deployed as portable devices or wireless sensor networks (WSN) to cover a large area in buildings [11–15]. Among the portable SPRi sensing devices, Guner et al. reported a smartphone-based SPRi biodetection platform. The device was composed of a green LED, a fiber optical cable, a bimetallic SPR sensor chip, a smartphone with a camera collecting the reflection from the sensor chip, and other beam shaping elements [15]. Though a resolution of 4.12 × 10^−5^ refractive index unit (RIU) was reported in this work, further application of the platform was hindered by the camera design updates in the smartphone and arbitrary bending of the fiber. Different from the reported portable devices, deployment of WSN is not dependent on the performance of the sensor, and does not even require the sensor itself to be mobile. Besides, WSN allows information to be collected and presented over a larger area, and the network transmission performance can be optimized by adjusting configuration parameters [11–14]. To deploy WSN in practice, we need to consider two factors. The first is the complexity of WSN, which is highly related to resource allocation and energy consumption [16]. In our previous work, the fractal dimension was used to evaluate the structural complexity of WSN [17]. The second is the transmission success rate, which is the key parameter in the evaluation of the network performance and user experience [18].

It is noteworthy that two factors need to be considered comprehensively in the performance optimization of both the plain silver SPRi sensor design and WSN deployment, which is multi-objective discrete optimization problems [19–21]. To solve such problems, various multi-objective optimization (MOO) algorithms have been reported, which can be divided into two main ways [22, 23]. The first type of the MOO algorithm can be categorized as the scalarization method. In this type of method, we can either combine all the individual objective functions into a composite function by weighting each objective or move all but one objective to a constraint set by setting a constraint value for each objective. In both of the choices, we can pursue a single solution considering all the objectives as the output of the optimization [24]. The second type of the MOO algorithm is known as the Pareto method. The output of the method is a set of single solutions, i.e., the Pareto optimal solution set. When we move from one solution to another in the set, a gain of one objective can be obtained at the cost of loss in another object [25]. Based on our previous works, we found that all the aforementioned performance factors of both the plain silver SPRi sensor and WSN cannot be expressed in individual objective functions, thus the MOO algorithms in the category of the Pareto method are the preferred choices in the performance optimization of both the sensor and the network. Due to its ability to find several solutions of the Pareto optimal solution set in one run with less dependency on the shape or continuity of the Pareto front in the whole process, the multi-objective genetic algorithms (MOGAs) have been widely used in mechanical engineering, industrial processes, and other intelligent decision-making fields [26, 27]. Genetic algorithms are search algorithms inspired by natural evolutionary theory. By mimicking the process of natural selection, crossover, and mutation, genetic algorithms can provide high-quality solutions in non-convex, discontinuous, and multimodal spaces to a variety of problems involving search, optimization, and learning [22]. MOGAs have been reported in the optimization of plasmonic structures and WSN performances [28,29]. In the optimization of plasmonic structures, Kim and Jung maximized the figure of merit (FOM) of the plasmonic curve and peak transmission power simultaneously by optimizing the slit width and height [28]. In the performance optimization of WSN, key factors, such as coverage, lifetime, energy consumption, and reliability, can be optimized simultaneously according to Fei et al. survey [29].

To enhance the DWR and PD value of the plain silver SPRi sensor, and improve the complexity and transmission success rate of the sensor-based WSN, we reported optimization of the silver SPRi sensor node-based WSN in this work. At the node level, we measured ellipsometer data of the silver SPRi sensor and calculated thickness-refractive index relations of different metals in the sensor. We then established two objective functions of DWR and PD of the sensor at different combinations of gold and silver thicknesses by using Kriging models. Afterward, we carried out the MOGA using the Pareto optimality. At the network level, we calculated the information dimension as complexity and the transmission success rate of WSN at different combinations of the number of nodes and transmission failure probability of nodes. We also established two objective functions of the two factors by Kriging models and carried out a similar MOGA algorithm. The results show that the performance parameters of both the plain silver SPRi sensor and WSN can be optimized by the Pareto optimal solution set obtained by MOGA. This optimization can not only help us to pursue the optimal choice of some certain performances of the sensor and the network but also assist us in making optimal decisions in practical sensor production and WSN deployment.

## 2. Methods

The work of the plain silver SPRi sensor-based WSN design and implementation includes three parts as in Figure 1: establishing objective functions of DWR and PD with the gold and silver thicknesses as variables by using the Kriging model, optimizing the film thicknesses by the MOGA algorithm, and optimizing the number of nodes and the hop count of WSN after setting up the objective functions of complexity and the transmission success rate. The calculation program was developed on the Python 3.7 platform on a personal computer with an Intel Core i7 2.8 GHz CPU and 16 GB RAM running the Windows 10 Ultimate operating system.

### 2.1. Optimization of Gold and Silver Thicknesses by MOGA

We used a spectroscopic ellipsometer (Sentech SE850DUV, SENTECH Instruments GmbH, Germany) to measure the intensity and phase of reflection from the sensor surface, and fitted the refractive indices of gold and silver films under different thickness conditions using the effective media approximation (EMA) compensated the Tauc-Lorentz (TL) model in commercial software WINELII according to the different elemental ratios of the gold and silver film layers [30]. Afterward, polynomial fitting was used to establish the correspondence between the refractive indices and thicknesses of gold and silver films at a wavelength of 660 nm, respectively. We then used the second-order universal Kriging (UK) interpolation method to establish the relationship between DWR, PD (Figure 2), and the gold and silver thicknesses based on the Jones transmission matrix, respectively, and used MOGA to find the Pareto optimal solution for gold and silver thicknesses with the optimization of the two indexes as the objective [28].

### 2.2. Improvement of Complexity and the Transmission Success Rate of WSN

Based on our previous work, we calculated both the information dimension and the transmission success rate of plain silver SPRi sensor-based WSN by the data transmission probability fractal model (PFM) with the number of nodes and transmission failure probability of nodes as variables [11,31]. Then, we established the objective functions of the two parameters by applying the second-order UK interpolation to the calculated data. After the MOGA optimization, we obtained a Pareto optimal solution set of the number of nodes and the hop count and validated the improvement of complexity and the transmission success rate.

## 3. Results and Discussion

### 3.1. Establishment of the Refractive Index-Thickness Models of Gold and Silver Films

According to our previous work, we fabricated the plain silver SPRi sensor of gold thickness ranging from 0.5 nm to 2.5 nm, and silver thickness ranging from 40 nm to 60 nm for spatial elemental distribution under transmission electron microscopy (TEM) [30]. A thicker silver film provides more atoms as the diffusion source and a longer fabrication process allowing the silver atoms to cross the gold-silver boundary, resulting in a higher elemental ratio in the gold layer. Thus, as shown in Figure 3(a), when the gold film becomes thinner and the silver film becomes thicker, the gold element ratio in the gold film side of the gold-silver boundary decreases dramatically. In the contrast, the gold film is much thinner compared with the silver film, which cannot provide sufficient gold atoms diffusing across the gold-silver boundary, resulting in an elemental ratio of less than 10% in the silver film as shown in Figure 3(b).

In the ellipsometer measurement, intensity and phase data of reflection from the silver surface of the sensor were collected for data fitting. Considering the thin gold film was covered by the thick silver film, we did not fit the refractive index of the gold film, but calculated the index value by the EMA method instead [32]. During fitting the refractive index of the silver film, the EMA compensated TL model can be described as in equations (1) and (2). In equation (1), *ε*_*i*_ and *ε*_*r*_ represent the real part and the imaginary part of the dielectric constant, respectively. *E*, *A*, *E*_*0*_, *Eg*, *C*, *P*, and *ε*_*r*_(∞) represent the energy of a photon, amplitude, peak transition energy, band gap energy, spreading correction parameter, Cauchy body value, and fitting correction parameter of the silver element, respectively. In equation (2), *G* represents the depolarization parameter of the silver element, and *ε* is the dielectric constant calculated by equation (1). *f*_*f*_ and *f*_*v*_ are the silver and gold element ratios in the silver film observed under TEM, and *n*_EMA_ is the effective refractive index of the silver film for the fitting work [33–35].

(1) $$\begin{array}{c} \varepsilon_{i}\left(E\right)=\frac{AE_{0}C{\left(E-E_{g}\right)}^{2}}{{\left(E^{2}-E_{0}^{2}\right)}^{2}+C^{2}E^{2}}\cdot \frac{1}{E},\varepsilon_{r}\left(E\right)=\varepsilon_{r}\left(\infty \right)+\frac{2}{\pi }P\int \frac{\xi \varepsilon_{i}\left(\xi \right)}{\xi^{2}-E^{2}}d\xi \;, \end{array}$$

(2) $$\begin{array}{c} f_{f}\frac{\varepsilon -n_{\text{EMA}}^{2}}{n_{\text{EMA}}^{2}+G\left(\varepsilon -n_{\text{EMA}}^{2}\right)}+f_{v}\frac{1-n_{\text{EMA}}^{2}}{n_{\text{EMA}}^{2}+G\left(1-n_{\text{EMA}}^{2}\right)}=0. \end{array}$$

Owing to the diffusion of gold atoms in silver film, the fitted imaginary part of the refractive index is smaller than the theoretical value of the silver bulk material in Figure 4(b). The small imaginary part of the refractive index can help increase the reflectivity of the metal surface, thus the measured reflection is higher than the fitted data, while the measured phase data can be fitted well in Figure 5. Besides, the real part of the refractive index is smaller than that of the theoretical value at the wavelength ranges from 500 nm to 750 nm in Figure 4(a), while the measured reflection is around 0.04 higher than the fitted data in the same range (Figure 5(a)). This phenomenon indicates that high reflectivity can affect the fitting accuracy of the real part of the refractive index [35].

We repeated the same ellipsometer measurement and curve-fitting work to the plain silver SPRi sensor of other gold and silver thicknesses, and calculated the relation between the refractive index at a wavelength of 600 nm and thickness of both the gold and silver films by polynomial fitting as in equation (3) [36,37]. For gold and silver, *f*_*f*_ (%) in equation (3) can be expressed as functions of gold thickness *d*_*g*_ (nm) and silver thickness *d*_*s*_ (nm) in equations (4) and (5), respectively. Because of the mutual diffusion between the gold and silver films during fabrication, the refractive index expressions of the metals contain the thicknesses of both films. It is noteworthy that the gold refractive index has a much stronger dependence on its thickness than silver, thus it is necessary to decrease the step of the gold thickness in the following second-order UK interpolation.

(3) $$\begin{array}{c} n_{\text{EMA}}^{2}=\varepsilon \cdot \left[{\left(1-\varepsilon \right)}^{2}f_{f}^{2}-5\left(1-\varepsilon \right)f_{f}+\varepsilon^{2}-3\varepsilon +3\right], \end{array}$$

(4) $$\begin{array}{c} f_{f}=17.64d_{g}-0.052d_{s}-3.94, \end{array}$$

(5) $$\begin{array}{c} f_{f}=-2.00d_{g}+0.16d_{s}+91.2. \end{array}$$

### 3.2. MOGA of Silver and Gold Thicknesses by Using Kriging Interpolation

Based on the aforementioned thickness-refractive index model of gold and silver films, we calculated the DWR and PD values at 660 nm according to the Jones transmission matrix at different gold and silver thicknesses [35]. Since DWR and PD can only be calculated according to Figure 2, the relation between the two parameters and these thicknesses are unknown functions and can be approximated by the second-order UK model according to reference [28]. In the approximation, the thickness steps of gold and silver films are 0.25 nm and 0.5 nm, respectively.

In Figure 6, we can see that the silver thickness is the key factor determining the incremental trend of DWR and PD rather than the gold thickness. Besides, the variations of DWR and PD do not appear to match each other well with the gold and silver thicknesses. Thus, both objective functions cannot be optimized by a single objective function, but need to be optimized for the Pareto optimal solution set for DWR and PD. Here, our problem can be expressed as equation (6), where *x* is a two-dimensional vector with components as the gold and silver thicknesses, and the *x*_*i*_^*L*^ and *x*_*i*_^*U*^ are the lower and upper bound of each variable, respectively. The multi-objective optimization problems are solved with a population size of 320, a crossover rate of 0.8, and a generation of 100 according to reference [28].

(6) $$\begin{array}{c} \text{Maximize DWR}\left(x\right)\text{ and PD}\left(x\right),\\ \text{subject to }x_{i}^{L}\leq x_{i}\leq x_{i}^{U},\;i=1,2. \end{array}$$

The optimized thicknesses of metallic films in the Pareto optimal solution set and corresponding objective function values listed in Table 1 show a similar trend to the data in Figure 6. For the different value of the gold thickness, the optimal silver thickness is around 58 nm, and the calculated DWR and PD varies less than 1%. This trend tells that the silver thickness is the most determinant of the performance of the silver SPRi sensor. We also notice that DWR and PD cannot be optimized at a single combination of gold and silver thicknesses. The combination no. 1 is desirable if we pursue a high DWR, while the combination no. 4 can be adopted if we need a large PD in the detection of bio-interactions occurring on the cell surface. Combination no. 9 may be chosen for practical manufacturing because a thick gold film may provide strong adhesion to the silver film [30].

### 3.3. Improvement of Complexity and the Transmission Success Rate of WSN

In previous work, we reported that increasing the number of nodes and decreasing the communication transmission failure probability of nodes can help to improve the transmission success rate [11]. However, the adjustment of the two factors has an impact on the information dimension of the network. The information dimension will become large if we increase the number of nodes or decrease the transmission failure probability of nodes [38]. Thus, we need to establish objective functions of the information dimension and the transmission success rate with the number of nodes and transmission failure probability of nodes as variables [39, 40]. Since the information dimension can only be calculated by a polynomial approximation, the aforementioned objective functions are unknown functions, which need to be approximated by the second-order UK model. In approximation with the hop count as 6, the range of the number of nodes is from 200 to 500 with 30 as a step, while the range of transmission failure probability is from 0.1 to 0.5 with 0.05 as a step [41, 42].

In Figure 7, the variations in the transmission success rate and the information dimension show an opposite trend with the variations in the number of nodes and transmission failure probability of nodes. Thus, both of the objective functions of the two performance parameters need to be optimized for the Pareto optimal solution set. Different from equation (6), our problem can be expressed as equation (7), where *x* is a two-dimensional vector with components as the number of nodes and the transmission failure probability of nodes. The multi-objective optimization problems are solved with a population size of 121, a crossover rate of 0.8, and a generation of 40.

(7) $$\begin{array}{c} \text{Maximize Success}\_\text{rate}\left(x\right)\text{ and Minimize Dimension}\left(x\right),\\ \text{subject to }x_{i}^{L}\leq x_{i}\leq x_{i}^{U},\;i=1,2. \end{array}$$

The optimized number of nodes and transmission failure probability of nodes in the Pareto optimal solution set and corresponding objective function values listed in Table 2 show a similar trend to the data in Figure 7. The information dimension and the transmission success rate cannot be optimized at a single combination of the two performance factors. The combination no. 1 is desirable if we pursue a small complexity of WSN, while the combination no. 5 can be adopted if a high transmission success rate is in urgent need. Combinations no. 2 and 3 may be chosen for deployment because both complexity and reliability are sufficient for practical usage.

## 4. Conclusion

In this work, we reported performance optimization of plain silver SPRi sensor-based WSN by using MOGA. In the optimization of the plain silver SPRi sensor, we chose the maximum values of DWR and PD as the optimization objective, and the thicknesses of gold and silver as variables to obtain the Pareto optimal solution set. In the optimization process, we established the refractive index-thickness models for both gold and silver, and calculated the DWR and PD values of the sensor with different gold and silver thicknesses by the Jones transfer matrix and Kriging interpolation. We found that DWR and PD cannot reach the maximum value simultaneously, but a trade-off can be made to get ambient results for both performance parameters. In the performance optimization of WSN, we chose the maximum value of the transmission success rate and the minimum value of the information dimension as the optimization objective, and the number of nodes and the transmission failure probability of nodes as variables. We also found that the aforementioned maximum and minimum values cannot be obtained simultaneously. By calculating the information dimension and the transmission success rate of each Pareto optimal solution, we obtained the number of nodes and transmission failure probability of nodes available for practical deployment of WSN. Besides, we can also provide the best solution for the optimization of some certain aforementioned performance parameters. The above results indicate that MOGA can be applied in simultaneous optimization of multiple parameters of sensors and networks in practical design, production, and deployment.

## Figures and Tables

**Figure 1:** Flowchart of the plain silver SPRi sensor wireless network design and implementation.

**Figure 2:** Principal illustration of (a) DWR and (b) PD in the plain silver SPRi sensor.

**Figure 3:** Gold element ratio in the (a) gold film side and (b) the silver film side of the gold-silver boundary under different gold and silver thicknesses.

**Figure 4:** Fitting and theoretical real part (a) and imaginary part (b) of the silver refractive index in the plain silver SPRi sensor.

**Figure 5:** Experimental (green) and fitting (red) results of (a) refraction and (b) phase data under ellipsometer measurement (gold: 2 nm, silver: 50 nm).

**Figure 6:** (a) DWR and (b) PD of the plain silver SPRi sensor after second-order UK interpolation.

**Figure 7:** (a) The transmission success rate and (b) the information dimension of WSN after second-order UK interpolation.

**Table 1:** Thicknesses of films and objective function values in the Pareto optimal set.

No.	Gold thickness (nm)	Silver thickness (nm)	DWR (%/°)	PD (nm)
1	0.5	58	365.503	459.314
2	0.75	58	364.880	465.498
3	1	58	363.922	455.690
4	1.25	57.5	364.661	466.833
5	1.5	57	363.475	458.975
6	1.75	58.5	364.500	460.193
7	2	58.5	363.944	458.526
8	2.25	57.5	363.239	459.284
9	2.5	58	363.591	459.689

**Table 2:** WSN performance factors and objective function values in pareto optimal set.

No.	Number of nodes	Transmission failure probability of nodes (%)	Information dimension	Transmission success rate (%)
1	260	0.45	1.95	84.5
2	320	0.35	2.53	88.1
3	350	0.3	2.81	90.8
4	380	0.2	3.12	93.0
5	440	0.15	3.60	96.3

## Data Availability

The data used to support the findings of this study are available from the corresponding author upon request.

## References

[1] Liu R., Wang Q., Li Q., Yang X., Wang K., Nie W. (2017). Surface plasmon resonance biosensor for sensitive detection of microRNA and cancer cell using multiple signal amplification strategy. *Biosensors and Bioelectronics*.

[2] Homola J. (2008). Surface plasmon resonance sensors for detection of chemical and biological species. *Chemistry Review*.

[3] Bradner J. E., McPherson O. M., Koehler A. N. (2006). A method for the covalent capture and screening of diverse small molecules in a microarray format. *Nature Protocols*.

[4] He L., Pagneux Q., Larroulet I. (2017). Label-free femtomolar cancer biomarker detection in human serum using graphene-coated surface plasmon resonance chips. *Biosensors and Bioelectronics*.

[5] Xia L., Yin S., Gao H., Deng Q., Du C. (2011). Sensitivity enhancement for surface plasmon resonance imaging biosensor by utilizing gold-silver bimetallic film configuration. *Plasmonics*.

[6] Chen S., Lin C. (2016). High-performance bimetallic film surface plasmon resonance sensor based on film thickness optimization. *Optik*.

[7] Li C. T., Yen T. J., Chen H. F. (2009). A generalized model of maximizing the sensitivity in intensity-interrogation surface plasmon resonance biosensors. *Optics Express*.

[8] Cheng Z., Wang Z., Gillespie D. E. (2015). Plain silver surface plasmon resonance for microarray application. *Analytical Chemistry*.

[9] Wang Z., Cheng Z., Singh V. (2014). Stable and sensitive silver surface plasmon resonance imaging sensor using trilayered metallic structures. *Analytical Chemistry*.

[10] Homola J., Piliarik M., Wolfbeis O. S. (2006). *Springer Series on Chemical Sensors and Biosensors*.

[11] Wang Z., Wang M. (2021). Wireless network of silver film lysozyme aptasensor based on fractal measurement. *Security and Communication Networks*.

[12] Zhan C., Zeng Y., Zhang R. (2018). Energy-efficient data collection in UAV enabled wireless sensor network. *IEEE Wireless Communications Letters*.

[13] Wang B., Gu X., Ma L., Yan S. (2017). Temperature error correction based on BP neural network in meteorological wireless sensor network. *International Journal of Sensor Networks*.

[14] Jain S., Nehra M., Kumar R. (2021). Internet of medical things (IoMT)-integrated biosensors for point-of-care testing of infectious diseases. *Biosensors and Bioelectronics*.

[15] Guner H., Ozgur E., Kokturk G. (2017). A smartphone based surface plasmon resonance imaging (SPRi) platform for on-site biodetection. *Sensors and Actuators B: Chemical*.

[16] Ndiaye M., Hancke G. P., Abu-Mahfouz A. M. (2017). Software defined networking for improved wireless sensor network management: a survey. *Sensors*.

[17] Wang Z., Zhou Y., Bajenaid A. S., Chen Y. (2022). Design of wireless sensor network using statistical fractal measurements. *Fractals*.

[18] Nayak S., Blumenfeld N. R., Laksanasopin T., Sia S. K. (2017). Point-of-Care diagnostics: recent developments in a connected age. *Analytical Chemistry*.

[19] López-Muñoz G. A., Estévez M. C., Vázquez-García M. (2018). Gold/silver/gold trilayer films on nanostructured polycarbonate substrates for direct and label-free nanoplasmonic biosensing. *Journal of Biophotonics*.

[20] Christodouleas D. C., Kaur B., Chorti P. (2018). From point-of-care testing to eHealth diagnostic devices (eDiagnostics). *ACS Central Science*.

[21] Liu Q., Li X., Liu H., Guo Z. (2020). Multi-objective metaheuristics for discrete optimization problems: a review of the state-of-the-art. *Applied Soft Computing*.

[22] Gunantara N., Ai Q. (2018). A review of multi-objective optimization: methods and its applications. *Cogent Engineering*.

[23] Konak A., Coit D. W., Smith A. E. (2006). Multi-objective optimization using genetic algorithms: a tutorial. *Reliability Engineering & System Safety*.

[24] Jia J., Fischer G. W., Dyer J. S. (1998). Attribute weighting methods and decision quality in the presence of response error: a simulation study. *Journal of Behavioral Decision Making*.

[25] Deb K., Datta R. (2012). Hybrid evolutionary multi-objective optimization and analysis of machining operations. *Engineering Optimization*.

[26] Pereira J. L. J., Oliver G. A., Francisco M. B., Cunha S. S., Gomes G. F. (2022). A review of multi-objective optimization: methods and algorithms in mechanical engineering problems. *Archives of Computational Methods in Engineering*.

[27] Cerda-Flores S. C., Rojas-Punzo A. A., Napoles-Rivera F. (2022). Applications of multi-objective optimization to industrial processes: a literature review. *Processes*.

[28] Kim K. Y., Jung J. (2017). Multiobjective optimization for a plasmonic nanoslit array sensor using Kriging models. *Applied Optics*.

[29] Fei Z., Li B., Yang S., Xing C., Chen H., Hanzo L. (2017). A survey of multi-objective optimization in wireless sensor networks: metrics, algorithms, and open problems. *IEEE Communications Surveys & Tutorials*.

[30] Wang Z., Wang Y., Wang M., Zheng Q. (2022). Analysis of adhesion strength between silver film and substrate in plain silver surface plasmon resonance imaging sensor. *Sensors and Materials*.

[31] Fan C., Dong T., Wen Z., Wu Q. A low energy algorithm of wireless sensor networks based on fractal dimension.

[32] Christy R. W. (1972). Optical constants of the noble metals. *Physical Review B*.

[33] Zhong C., Ballantine K. E., Kervick C. (2016). Mapping of surface plasmon dispersion in thin Ag–Au layered composite films. *Journal of the Optical Society of America B*.

[34] Jiang Y., Pillai S., Green M. A. (2016). Grain boundary effects on the optical constants and Drude relaxation times of silver films. *Journal of Applied Physics*.

[35] Peña-Rodríguez O., Caro M., Rivera A., Olivares J., Perlado J. M., Caro A. (2014). Optical properties of Au-Ag alloys: an ellipsometric study. *Optical Materials Express*.

[36] Dong J., Lu R. (2018). Characterization of weakly absorbing thin films by multiple linear regression analysis of absolute unwrapped phase in angle-resolved spectral reflectometry. *Optics Express*.

[37] Wang Z., Diamond J. J., Hou R. (2011). An accurate and precise polynomial model of angular interrogation surface plasmon resonance data. *Sensors and Actuators B: Chemical*.

[38] Wang J., Gao Y., Liu W., Sangaiah A., Kim H. J. (2019). An improved routing schema with special clustering using PSO algorithm for heterogeneous wireless sensor network. *Sensors*.

[39] Song C., Havlin S., Makse H. A. (2005). Self-similarity of complex networks. *Nature*.

[40] Kuo Y. W., Li C. L., Jhang J. H., Lin S. (2018). Design of a wireless sensor network-based IoT platform for wide area and heterogeneous applications. *IEEE Sensors Journal*.

[41] Wei D., Wei B., Hu Y., Zhang H., Deng Y. (2014). A new information dimension of complex networks. *Physics Letters A*.

[42] Khasawneh A., Latiff M. S. B. A., Kaiwartya O., Chizari H. (2018). A reliable energy-efficient pressure-based routing protocol for underwater wireless sensor network. *Wireless Networks*.

